RETRACTED

# Effects of thermal aging atmospheres on oxidation activity, element composition and microstructure of diesel soot particles

**DOI:** 10.1039/d3ra05340g

**Published:** 2023-10-13

**Authors:** He Huang, Zifei Ni, Wenkai Wang, Heng Chen

**Affiliations:** a School of Traffic Engineering, Nanjing Vocational University of Industry Technology Nanjing 210046 China 2018100903@niit.edu.cn +86-025-85864356

## Abstract

As an emission control device for diesel engines, DPF plays an important role in reducing particulate matter emissions. The research work on soot thermal aging will help optimize DPF regeneration strategies, improve regeneration efficiency, and promote the progress of engine emission control technology. In order to explore the influence of thermal aging under different atmospheres on particle physicochemical characteristics from diesel engines, the oxidation activity of soot particles after different thermal aging were evaluated by thermogravimetric analysis (TGA) and pyrolysis kinetics calculation, and the distribution of functional groups and elemental composition on the soot surface were investigated by FT-IR and XPS analysis. Additionally, the microstructure and graphitization degree of basic carbon with O_2_/NO_2_ aging were analyzed by HRTEM technology. The results show that the ignition temperature and activation energy of soot significantly increase after thermal aging, and their lowest values are 569 °C and 165.29 kJ mol^−1^ in O_2_/NO_2_/N_2_ atmosphere, respectively. The branching degree and content of hydrocarbon functional groups on the soot surface decrease after thermal aging, and the relative content of hydrocarbon functional groups with NO_2_ participating in thermal aging is the highest. The content of O element on the soot surface decreases after thermal aging, and the maximum O/C molar ratio of soot particles after thermal aging in O_2_/NO_2_/N_2_ atmosphere is 0.15. After thermal aging, the hybridization degree of carbon atoms and the content of –C–OH and –C=O functional groups on the soot surface decrease. The content of –C–OH functional group decreases to 0.21% and 0.53% respectively after the addition of O_2_ and NO_2_ in the thermal aging atmosphere, while the content of –C=O functional group increases to 4.98% and 5.98% respectively. In addition, the layer spacing and microcrystalline curvature of basic carbon particles decrease after thermal aging, however, the microcrystalline size and the graphitization degree increase.

## Abstract 2

As an emission control device for diesel engines, DPF plays an important role in reducing particulate matter emissions.

## Introduction

Under the current international situation, the demand for global energy is growing very rapidly.^1^ With the increasing scarcity of global oil resources, the issue of fossil fuel consumption is becoming increasingly prominent.^2–4^ Diesel engines are widely used as power units in fields such as transportation, industry, and agriculture.^5^ However, the exhaust emissions from diesel engines have an undeniable impact on human health and climate change.^6,7^ The exhaust components of diesel engines mainly include carbon dioxide (CO_2_), carbon monoxide (CO), nitrogen oxides (NO_*x*_), hydrocarbons (CH), and particulate matter (PM).^8,9^ The existing technical means to reduce engine emissions are mainly divided into internal purification technology and external purification technology. The internal purification technology includes the use of low-temperature combustion mode, exhaust gas recirculation, and alternative fuels.^10,11^ The external purification technology mainly includes diesel oxidation catalysts (DOCs), diesel particulate filters (DPFs), selective catalytic reduction (SCR), and so on. Diesel particulate matter mainly contains soot, soluble organic fraction (SOF) sulfate,^12^ and soot is the primary constituent of diesel particulate matter, constituting ap-proximately 60% to 70% of its composition. Soot particles are usually produced in large quantities at high loads, and the formation conditions are local high temperature and hypoxia inside the cylinder. Diesel particulate filter (DPF) is the most effective device to reduce particle emissions, which can be reduced to 10% after treatment.^13,14^ With the amount of soot captured increases, the pressure drop of the DPF will rise, leading to a decline in engine combustion performance and power output. Therefore, it is necessary to periodically oxidize and regenerate the soot accumulated in the DPF.^15^ DPF mainly has active and passive regeneration modes: the active regeneration is to rise the temperature in DPF, so that the soot accumulated in the channel reaches a certain temperature and oxidizes; and the passive regeneration is to coat the catalyst with better activity on the support, so as to reduce the oxidation characteristic temperature of soot particles. In addition to the environmental factors of the oxidation regeneration reaction of soot, the physical and chemical properties of soot also have a decisive impact on the regeneration of DPF. Because DPF regeneration has a periodic feature, soot will be deposited in DPF for a period of time before regeneration, and the diesel exhaust temperature and composition will change in real time with the working conditions. Under the influence of the intricate high-temperature exhaust conditions, the physical and chemical properties of soot will be affected, resulting in the complex oxidation characteristics. This process is called “thermal deactivation’’ of carbon components,^16^ also known as the thermal aging process of diesel soot.^17^ It can be seen that it is of practical significance for the study of DPF regeneration process to explore the changes of physical, chemical and oxidative properties of soot during thermal aging. The oxidation activity of diesel soot is closely related to its physical and chemical characteristics. Diesel soot is composed of disordered soot particles inside, while the outside is a clear graphitized structure. A significant presence of active functional groups can be observed at the surface of soot, particularly at the edges or defect sites. Functional groups are specific atomic groups attached to the soot surface, and are active substances produced during the oxidation process of soot, including oxygen-containing functional groups and hydrocarbon functional groups, which play certain specific roles in the soot oxidation process.^18,19^

RETRACTED

Domestic and foreign scholars have analyzed the physical and chemical characteristics of soot particles by various means. Ferrari *et al.*^20^ found that the *I*_D_/*I*_G_ ratio can be used to evaluate the graphitized structure of soot particles in Raman spectrum of soot, while the small *I*_D_/*I*_G_ represents a high degree of graphitization, and the structure of soot is stable and not easy to oxidize. Cain *et al.*^21^ found that when there are oxygen-containing groups on the surface of carbon smoke, its oxidation activation energy decreases. As oxidation progresses, the activation energy of all soot samples is very similar when oxygen-containing groups are lost, indicating that the presence of oxygen-containing groups has no lasting effect on sample oxidation. Wang *et al.*^22^ determined the types of functional groups by studying the distribution characteristics of soot particles possess various functional groups on their surface in premixed flame, and found that the sur-face of the soot particles contains aliphatic hydrocarbon functional groups as well as aromatic hydrocarbon functional groups, C=C non-oxygen functional groups and –C–OH and –C=O oxygen functional groups, and the content regarding aliphatic hydrocarbon is relatively high. Meng *et al.*^23^ studied the effect of heating rate on the oxidation performance of soot through thermogravimetric experiments and found that the reactivity of soot increases with the increase of heating rate. Pena *et al.*^24^ found that with the increase of fuel flow, the transverse size of the aromatic layer in the soot decreases, the concentration of aliphatic and oxygen-containing groups decreases, and the concentration of aromatic groups increases. Some studies also indicate that the oxidation characteristics of soot largely depend on the microstructure of the initial soot state. E. *et al.*^25^ found that operating conditions can change the distribution of temperature field inside the particle trap, directly affecting the regeneration process of the trap. In addition to the increase in O_2_ concentration and exhaust gas flow rate, the initial amount of soot particles also affects the regeneration process. When the initial mass of soot is less than the critical value of the trap, the regeneration speed will decrease. Fang *et al.*^26^ studied the effect of operating parameters on the regeneration performance of DPF using a regeneration experimental bench and proposed that under a soot loading rate of 2.5 g L^−1^, the regeneration efficiency increases with the increase of regeneration flow rate. Soltani *et al.*^27^ studied the oxidation of NO_2_ non catalytic soot by water vapor, and the study showed that water vapor has a promoting effect on the oxidation of soot. In addition, under specific conditions, NO_2_, water, and O_2_ have a synergistic effect on the oxidation of soot. Zhao *et al.*^28^ found that higher relative concentration of C–S bond corresponds to shorter soot streak length, and the relative amount of –SH and C–S bonds can improve the oxidation reactivity of soot. Guo *et al.*^29^ studied the carbon skeleton of soot through Raman spectroscopy, and found that the breakdown of soot was due to the fracture of chemical bonds on the bridging site, and the oxidation process was dominated by the oxygen-containing functional groups located at the outer region of the soot particles. However, there are relatively few studies on the surface of soot particles conversion and oxidation reaction of diesel soot particles during thermal aging process at home and abroad.

RETRACTED

The oxygen-containing functional groups on the surface of soot have a significant impact on the oxidation characteristics of soot. Thermal aging can cause changes in the number and structure of functional groups on the surface of soot, thereby affecting the surface properties and oxidation reaction activity of soot. There is currently limited research on the reaction mechanism and effects of O_2_ and NO_2_ oxidation media during the thermal aging process of soot. In order to better utilize the NO_2_ component in the exhaust, promote the soot oxidation, and achieve the regeneration process of DPF, it is necessary to conduct in-depth research on the physicochemical characteristics changes of diesel soot after thermal aging in O_2_ and NO_2_ atmospheres. Therefore, this study investigated the effects of thermal aging under different atmospheres on various functional groups on the surface of soot and the oxidation characteristics of soot. Firstly, the collection and thermal aging pre-treatment of diesel soot particles are carried out based on the low speed and high load conditions with high smoke emission. Secondly, the oxidation characteristics of different soot samples are studied by thermogravimetry analysis (TGA) and pyrolysis kinetics calculation. Thirdly, the distribution of functional groups and element composition on soot surface are analyzed through Fourier transform infrared (FT-IR) and X-ray photoelectron spectroscopy (XPS) tests. Finally, the layer spacing, microcrystal-line size and microcrystalline curvature of soot carbon are measured by high-resolution transmission electron microscope (HRTEM), and then the changes of the microstructure and graphitization degree of basic carbon particles with O_2_/NO_2_ aging are studied.

## Experimental

### Soot samples collection and thermal aging treatment

The experiments were carried out on a turbocharged diesel engine with four cylinders, which was operated for 2 h at low speed and high load. The exhaust particles were sampled with the self-made device as shown in Fig. 1. Then the organic solvent ethanol was selected to dilute and wash the particles, and put them into the ultrasonic cleaner to oscillate and disperse. Remove the surface solution containing SOF and dry it to obtain the soot sample for the test.

**Fig. 1:** Soot collection device.

The thermal aging device shown in Fig. 2 was used to study the effects of thermal aging on diesel soot samples under different conditions. The experimental system mainly consists of a simulated atmosphere device and a heating device. The simulated diesel exhaust is diluted and mixed with O_2_/NO_2_/N_2_. The mixture enters the soot thermal aging reactor to participate in the soot thermal aging process. The heating furnace is KJ-T1200-S5060LK model of KEJIA Company. The test temperature and time are set by automatic programming, and the experimental process is monitored by computer receiving sensor signals.

**Fig. 2:** Schematic diagram of thermal aging treatment system.

The exhaust temperature at most operating conditions of diesel engines ranges from 473 to 723 K.^30^ The volume fraction of O_2_ in diesel exhaust is about 10%, while the volume fraction of NO_2_ after diesel oxidation catalyst (DOC) is between 0.01% and 0.04%. Therefore, the volume fractions of O_2_ and NO_2_ in the thermal aging atmosphere are 10% and 0.04%, respectively. Soot samples after thermal aging under different atmospheres are recorded as DS-1, DS-2 and DS-3, while untreated reference samples are recorded as DS-0, as shown in Table 1. The duration of each thermal aging is 80 min, the diameter of quartz tube used is 6 mm, and the gas flow speed is 200 mL min^−1^. After the test, soot sample should be placed in a dry sealed container to ensure the accuracy for the next characterization. The blast drying oven is used as the drying apparatus in this study. The drying temperature is 110 °C and the drying time is 24 hours.

RETRACTED

**Table 1:** Parameters of thermal aging atmosphere

Soot samples	O_2_ (%)	N_2_O (ppm)	N_2_ (ppm)
DS-1	0	0	100
DS-2	10	0	90
DS-3	10	400	90

## Methods

The oxidation characteristics of diesel soot after thermal aging in different atmospheres are analyzed by thermogravimetry (TG) test. The model of thermogravimetric analyzer selected in TG test is TGA/DSC1 from METTLER Company, Switzerland. Its function is to measure the change of mass with temperature during physical and chemical changes such as evaporation, pyrolysis and oxidation of substances. After the thermal aging test, about 5 mg of soot sample is weighed and put into the thermogravimetric analyzer. 10% O_2_ and 90% N_2_ are selected as the working gas and mixed into the reactor, and N_2_ is chosen as the gas for protection. Gases flow is fixed at 100 mL min^−1^. Meanwhile, programmed reaction intermission was set between 353.15 K and 1073.15 K, and the heating rate was controlled at 30 K min^−1^.

Three oxidation characteristic temperatures are selected. The soot ignition temperature (*T*) refers to the temperature at which a 10% mass loss occurs, while the peak combustion temperature (*T*_m_) refers to the temperature at which the peak mass loss is observed, and the burnout temperature (*T*_f_) is the temperature corresponding to the mass loss of 90%. The soot oxidation characteristics were studied by oxidation kinetics analysis method, and TG test data were analyzed to calculate the activation energy of soot oxidation reaction.^31^ The activation energy of soot oxidation reaction was calculated by Coast–Redfern integration method. The formula for calculating the weight loss rate of soot is as follows:1where, *m*_o_ is the total mass of soot, and *m* is the mass corresponding to the current temperature *T*.

The oxidation rate is expressed as:^32^2

3 *f*(*α*) = (1 − *α*)^*n*^

where, *α* is weight loss rate of soot, (%); *A* is pre-exponential factor, s^−1^; *E* is the activation energy of reaction, kJ mol^−1^; *R* is the universal gas constant, 8.314 × 10^−3^ (kJ K^−1^ mol^−1^); *f*(*α*) is the reaction function, *n* is reaction order.

Integrate both sides of formula (2):4

Because *E*/*RT* ≫ 1, the above formula can be simplified as:5where, *T* is the thermodynamic temperature, K; *β* is the heating rate, K min^−1^; *E* is the activation energy, J mol^−1^. *E* of soot can be calculated by linear fitting.

RETRACTED

FT-IR (Thermo Scientific Nicolet iS5) was used to analyze the relative content of hydrocarbon functional groups. The scanning resolution is 0.1 cm^−1^ and the scanning range is 0–4000 cm^−1^. The background calibration uses high-purity KBr. The hydrocarbon functional groups in diesel soot typically exhibit absorption bands in the range of 2700–2975 cm^−1^. The presence of phenolic aromatic rings or fused rings can be identified by characteristic peaks around 1620 cm^−1^, indicating the presence of carbon–carbon bonding.

The X-ray photoelectron spectroscopy (XPS) technique was employed to analyze the elemental composition and oxygen-containing functional groups present on the surface of the soot particles. The C 1s binding energy of at 284.6 eV was used as an internal calibration using the casaXPS software. Light source is Al Kα X-ray, power 0.3 kW, limit energy resolution 0.43 eV, energy range 0–5000 eV, scanning step 1 eV.

HRTEM (Tecnai G2F30) was used to effectively observe the microstructure of soot samples, and the characteristic parameters of soot microstructure, such as layer spacing, microcrystalline size and microcrystalline curvature, were obtained. Electron micro-scope limit is 2.3 × 10^5^ times, the extreme voltage is 300 kV, and the point-line resolution can reach 0.15 nm.

## Results and discussion

### Thermogravimetric analysis (TGA)

Fig. 3 shows the TG and DTG curves of different soot samples. It can be seen from Fig. 3(a) that the mass loss of soot after thermal aging is significantly less than DS-0 at 80–547 °C. This is mainly because the content of substances easy to evaporate and oxidize in soot particles is significantly reduced due to thermal aging. With the gradual increase of temperature, the weight loss rate of soot increases significantly when the ignition temperature of soot is reached. When the temperature is raised to about 690 °C, the residual mass of soot is reduced to the minimum. Compared with DS-0, all kinds of aging make the weight loss curve of soot oxidation stage shift to the high-temperature region, and the change in the early stage of the oxidation process is more obvious. Compared with DS-1, DS-2 and DS-3, the weight loss curve shifts to the low-temperature region, while the weight loss curve of DS-3 is closer to DS-0. It can be found from Fig. 3(b) that the peak positions of soot combustion rate after different thermal aging are basically the same, which indicates that the influence of thermal aging is mainly situated at the initial stage of combustion of soot oxidation. It can be seen from Table 2 that the change of oxidation characteristic temperature primarily observed during the early oxidation stage of various soot samples. The change of *T*_*i*_ is more obvious, with the maximum difference of 13 °C, while the changes of *T*_m_ and *T*_f_ are relatively small, with the maximum difference of 5 °C and 3 °C respectively.

RETRACTED

**Fig. 3:** (a) TG and (b) DTG curves of soot samples after thermal aging.

**Table 2:** Oxidation characteristic temperatures of soot samples with thermal aging

Soot samples	*T*_*i*_ (°C)	*T*_m_ (°C)	*T*_f_ (°C)
DS-0	566	645	680
DS-1	579	649	681
DS-2	577	650	679
DS-3	569	646	680

The TG curve is analyzed and fitted to calculate the activation energy of soot. The fitting curve is shown in Fig. 4. Table 3 displays the oxidation kinetic parameters for the different samples, including the fitted equations for the different atmospheres and the corresponding activation energies of the thermal aging soot. It can be seen that the highest activation energy of thermal aging soot under N_2_ atmosphere is about 183.5 kJ mol^−1^. Compared with thermal aging soot under N_2_, the activation energy of soot is reduced by both O_2_ and NO_2_ in the thermal aging atmosphere. Among them, the activation energy of thermal aging soot under O_2_/NO_2_ atmosphere is the lowest, about 165.3 kJ mol^−1^. Combining Fig. 3 and Table 2, it can be found that this is because under O_2_/NO_2_ atmosphere, the weight loss rate of soot is the highest and the ignition temperature is the lowest. Under N_2_ atmosphere, the weight loss rate of soot is the lowest and the ignition temperature is the highest. Therefore, the changes in activation energy of thermal aging soot under different atmospheres correspond to TG curves and oxidation characteristic temperature trends.

**Fig. 4:** Fitting curves for oxidation activation energy of soot.

**Table 3:** Activation energy of soot samples after thermal aging

Soot sample	Fitting equation	*R* ^2^	Activation energy (kJ mol^−1^)
DS-0	*Y* = −19.425*x* + 7.494	0.968	161.5
DS-1	*Y* = −22.075*x* + 10.286	0.995	183.5
DS-2	*Y* = −21.935*x* + 10.175	0.990	182.4
DS-3	*Y* = −19.881*x* + 8.001	0.968	165.3

Research has shown that the thermal aging atmosphere has a significant impact on the oxidation characteristic temperature and reaction activation energy of soot, and its physicochemical properties after thermal aging are more complex. Therefore, the physical and chemical properties of soot after thermal ageing were next characterized.

### FTIR analysis

The exterior of diesel soot particles exhibits three types of functional groups: oxygen-containing functional groups (C–O, –C=O, and –C–OH), hydrocarbon functional groups (–CH_3_ and –CH_2_), and aromatic ring (C=C) functional groups.^33^Fig. 5 shows the infrared spectra of DS-0, DS-1, DS-2 and DS-3 soot samples. The observed pattern rules regarding various samples are generally constant, with principal distinction lying in the peak height and peak width of each peak, which indicates that there is no obvious difference in the types of functional groups on the surface regarding soot particles after thermal aging, and the variation primarily manifests in the relative proportions regarding distinct functional groups. Methoxy C–O usually shows absorption peaks in the wave number range between about 1100 and 1300 cm^−1^, with a distinct characteristic peak at 1080 cm^−1^, which is due to the stretching vibration of methoxy. There is a high and broad absorption peak at 3435 cm^−1^ in the wave number range of 3100–3700 cm^−1^, which is due to the presence of hydroxyl (–OH) functional groups on the surface of the oxidized soot. In the wave number range of hydrocarbon functional groups, two prominent characteristic peaks were observed at 2920 cm^−1^ and 2854 cm^−1^, which correspond to –CH_3_ and –CH_2_ of aliphatic asymmetric stretching vibration and symmetric stretching vibration respectively. The intensity of asymmetric stretching vibration of aliphatic hydrocarbon functional groups in soot is significantly higher, indicating aliphatic hydrocarbons in soot predominantly exist in short chains.^34^

RETRACTED

**Fig. 5:** Infrared absorbance spectrum of soot samples after thermal aging.

In order to evaluate the content of functional groups on the surface of diesel engines, the *I*_2920_/*I*_2854_ ratio of the peak heights at 2920 cm^−1^ and 2854 cm^−1^ is utilized to assess the degree of branching of hydrocarbon functional groups, and the *I*_2920_/*I*_1620_ ratio of peak heights at 2920 cm^−1^ and 1620 cm^−1^ is utilized to assess the proportion of aliphatic hydrocarbon functional groups in diesel soot.^35^ As can be seen from Fig. 6, compared with nonaged soot, the *I*_2920_/*I*_2854_ of soot decreases from 1.26 to 1.24, 1.20 and 1.19 respectively with thermal aging in different atmospheres, which indicates that the branching degree of hydrocarbon functional groups decreases after thermal aging. This is because the symmetry stretching vibration of –CH_2_ is relatively unstable, and it is easy to lose during soot thermal aging, thus reducing the branching degree and activity of hydrocarbon functional groups of soot. Compared with DS-1, the addition of O_2_ and NO_2_ in thermal aging atmosphere will further decrease the branching degree of the surface of soot particles containing hydrocarbon functional groups, but in general, different thermal aging atmospheres have little effect on the branching degree of hydrocarbon functional groups of soot. After thermal aging, the relative content of hydrocarbon functional groups on the surface of soot also decreases to varying degrees. The *I*_2920_/*I*_1620_ ratios of DS-1, DS-2 and DS-3 are 0.57, 0.45 and 0.51 respectively. Compared with DS-1, the decrease of DS-2 is more obvious due to the addition of O_2_, but with the addition of NO_2_, the hydrocarbon functional groups constitute the majority of functional groups on the surface of soot particles will rise again. This is because in the thermal aging process of soot, the C=C functional group is more stable than the hydrocarbon functional group,^36^ and the aliphatic hydrocarbon functional group on the surface of soot will undergo hydrogen atom stripping and thermal decomposition, so that the functional group structure is gradually oxidized and reduced.^37^ Generally, hydrocarbon functional groups mainly exist at the edge of the microcrystalline layer of soot particles, so their relative activity is high and they are easy to oxidize.^38^ The change in their content will also affect the oxidation activity of soot. Hydrocarbon functional groups cannot be generated during thermal aging. After further addition of NO_2_ in the thermal aging atmosphere, some of them will be decomposed into NO and O_2_, making the O_2_ concentration higher. At the same time, NO_2_ has stronger oxidation. This gas component has stronger oxidation effect on C=C functional groups than pure O_2_, which promotes more C=C functional groups to participate in the oxidation reaction, increases C=C consumption rate, and generates more oxygen-containing functional groups, thus resulting in an increase in the relative proportion of hydrocarbon functional groups.

RETRACTED

**Fig. 6:** Branching degree of hydrocarbon functional groups in soot samples after thermal aging.

### XPS analysis

Fig. 7 depicts the XPS full spectrum of soot particles after thermal aging in different atmospheres. Different soot samples have obvious peaks at 285 eV and 533 eV, which can be judged as C 1s spectrum peak and O 1s spectrum peak according to the appearance position. The soot surface is mainly composed of C and O elements. In addition, there are other elements in the soot, but due to the low content, the intensity is low when the XPS spectrum is taken, and no obvious peak is formed, which is difficult to be observed in the spectrum.

**Fig. 7:** XPS spectrum of soot samples after thermal aging.

By removing the background line in the full spectrum, the relative molar contents of C and O can be calculated. The relative content of O and C on the outside of non-aged soot particles is about 15.1% and 83.8% respectively. The molar ratio of O/C could be analyzed by their ratios. Fig. 8 presents the O/C molar ratio for various soot samples, and the O/C molar ratio of non-aged soot particles is 0.18. The oxygen element on the surface of soot particles after thermal aging decreases, and the oxygen element content of soot particles aged in O_2_/NO_2_ atmosphere is relatively the highest, about 0.15. This is because during the thermal aging process, the oxygen-containing functional groups will undergo pyrolysis and oxidation, which is mainly pyrolysis reaction in pure N_2_ atmosphere, resulting in a decrease in the content of O element on soot surface. Since the thermal aging temperature is far lower than the ignition temperature of soot particles, the soot will not undergo deep-seated oxidation reaction, and part of C will react with the oxidizing active gases O_2_ and NO_2_ to generate the intermediate product C (O) of soot oxidation. Compared with O_2_ atmosphere, the content of oxidizing active gases in NO_2_/O_2_ atmosphere is more, which is easier to react with soot and form relatively more C (O) intermediates, so that the content of O element detected in the soot sample is higher than that of other aged soot, which also facilitates the oxidative reaction of soot.

**Fig. 8:** The O/C ratio on the surface of soot samples after thermal aging.

In order to study the existing form of C element on the surface of soot particle, the peak of C element can be fitted by XPS peaks software, and the relative content of oxygen-containing functional groups and the hybridization degree of carbon atoms can be calculated by the fitting curve. The electrons outside a single atomic nucleus will be orderly arranged in different orbits according to certain rules. In a molecule, different atomic orbits will be recombined, which will affect the overall stability of the molecule. This process is called atomic hybridization. The hybrid forms of carbon atoms include sp^2^ hybrid and sp^3^ hybrid, which are commonly employed to assess the level of disorder in soot and to characterize its stability. A higher sp^3^ content indicates a greater degree of disorder in soot, whereas a higher sp^2^ content indicates a more ordered structure and greater stability of soot. Hence, the sp^3^/sp^2^ ratio is commonly utilized to directly serve as an indicator of the structural properties of soot in soot research.^39^

Fig. 9 shows the fitting curve of C 1s peaks of four soot samples. As depicted in the diagram, there are four forms of C atoms: sp^2^ hybrid, sp^3^ hybrid, hydroxyl (–C–OH) functional group and carbonyl (–C=O) functional group, which appear near 284.8 eV, 285.5 eV, 286.8 eV and 287.8 eV respectively. Therefore, the peak splitting of C 1s peaks is fitted into four characteristic peaks, corresponding to the above four C atom structures. The area of C 1s peak and four small characteristic peaks are calculated, the degree of disorder of soot is calculated by the proportion of the peak region corresponding to sp^2^ hybrid and sp^3^ hybrid, and the ratio of peak area of these two functional groups to the overall area of C 1s peak can be calculated by the relative content of –OH and –C=O.

RETRACTED

**Fig. 9:** Fitting curves of C 1s peaks of (a) DS-0, (b) DS-1, (c) DS-2 and (d) DS-3.

The soot surface is mainly graphitized, and disordered carbon mainly exists at the edge of graphitized structure. In addition, the microstructure of disordered carbon is fine and disordered with more functional groups at the edge. These structures are un-stable and easy to be oxidized. Therefore, they a positive role in the oxidation process of soot, and soot with high degree of disorder is more likely to react in the oxidation process. Fig. 10 shows the degree of carbon atom hybridization of different soot samples. After thermal aging, the degree of disorder of carbon atoms decreases. The sp^3^/sp^2^ ratio of non-aging soot is 0.51, and the sp^3^/sp^2^ ratio of other aged soot is 0.37, 0.32 and 0.31 respectively. Compared with soot after thermal aging in N_2_ atmosphere, the ratio in O_2_ and NO_2_ atmosphere further decreases. Compared with sp^2^ hybrid carbon atom, sp^3^ hybrid carbon atom has higher activity and is easier to be consumed. High temperature will change the microstructure of soot,^40^ consume part of functional groups on soot surface, as well as most of ordered structure residues. These factors comprehensively lead to a decline in the chaos degree regarding soot after thermal aging.

**Fig. 10:** Carbon atom hybridization on the surface of soot samples after thermal aging.

Fig. 11 shows the relative content of oxygen-containing functional groups on the surface of soot after thermal aging in different atmospheres. Compared with the non-aging soot, the proportion of –C–OH functional groups on the surface of the N_2_-aged soot decreases to 11.52%. When the atmosphere is O_2_ and NO_2_/O_2_, the proportion of –C–OH significantly further decreases, and most of them are consumed during the thermal aging process. This shows that during the thermal aging process in pure N_2_ atmosphere, the consumption of –C–OH functional group is less, but the –C–OH functional group is easy to react with O_2_ and NO_2_. At the same time, there is no H element in the atmosphere, so the functional group containing H element will not be formed on the soot surface during the thermal aging. Most of –C=O thermally aged in N_2_ atmosphere is consumed, and the content obviously decreases to 0.46%, which indicates that the –C=O functional group is easily consumed in the non-oxidation process. However, after thermal aging in O_2_ and NO_2_/O_2_ atmosphere, the content of –C=O functional groups *t* increases by 4.52% and 5.52%. The –C=O functional groups will react with O_2_ and NO_2_ to be consumed, so the increase of the content of –C=O functional groups indicates that the detected part of –C=O functional groups are formed during the thermal aging process, which is attributed to the oxidation activity of O_2_ and NO_2_, and the incomplete oxidation reaction occurs with soot. Meanwhile, the formation rate of –C=O functional groups is higher than the consumption rate during the thermal aging process, which also leads to an increase in the detectable O element content on soot surface. The increased O element mainly comes from the generated –C=O functional groups.^41^

RETRACTED

**Fig. 11:** Relative content of functional groups on the surface of soot samples after thermal aging.

### HRTEM analysis

Fig. 12 displays the HRTEM images of soot particles, which clearly and comprehensively reflects the microstructure of non-aged soot and soot after thermal aging in O_2_/NO_2_ atmosphere. The size of soot particles is about 30 nm, and both soot samples are “shell core” structure, which is composed of shell and core. The “shell” is a micro-crystalline layer stacked in multiple layers, and it can be observed by the naked eye that the length is relatively consistent and stacked in a relatively regular order. The “core” is composed of microcrystals with no fixed length and shape, which is messy and disordered. This shell–core structure is a balanced and relatively stable structure, which is formed by the orientation elastic deformation of polycyclic aromatic hydrocarbon lamellae exceeding the crystal-free energy under high temperature conditions. At the same time, soot particles have two forms: “single-core” and “multi-core”. The “multi-core” structure is formed by the rapid collision and condensation of small particles before they grow into large particles.^42^

**Fig. 12:** HRTEM images of (a) DS-0 and (b) DS-3 soot particles.

It can be observed from Fig. 12(b) that the edges of non-aged soot particles are more blurred, and more amorphous soot structures can be found. The “shell–core” structure is more obvious than that after thermal aging, and the arrangement of internal microcrystalline structures is more disordered. The thermal aging process makes the structure of soot particles change. The microstructure regarding soot particles is related to oxidation activity. The core of soot particles is easier to be oxidized because of its disordered structure, and the shell structure is more stable and difficult to be oxidized, so the soot with high graphitization degree has lower activity. In order to more intuitively characterize the effect of thermal aging, the three main characteristic parameters of soot microstructure, namely, the layer spacing, microcrystalline size and microcrystalline curvature, were measured and the distribution histogram was drawn.

RETRACTED

Fig. 13(a) shows the distribution histogram of the layer spacing. It can be found that the layer spacing of all soot samples is between 0.26 nm and 5.0 nm, which is consistent with the results of Christensen *et al.*^43^ The peak ratio of layer spacing of the basic carbon particles of the two soot samples is 0.34 nm–0.38 nm, it can be observed intuitively that the average layer spacing of non-aged soot particles is greater than that of thermal aging soot particles. When making statistics on the micro-size parameters of basic carbon particles, the commonly used algorithm will screen out the microcrystals whose size is less than the minimum value, because these tiny soot microcrystals are difficult to distinguish from the amorphous ones due to their similar structures in the statistical process. The determination of the minimum microcrystalline size is different in various studies, and 0.55 nm is selected as the minimum value in this study. Fig. 13(b) shows the microcrystalline size of carbon particles in soot samples. The microcrystalline size of the various soot samples ranges from 0.55 nm to 5.05 nm, as evident from the observations. The peak proportion of the crystallite size of non-aged soot particles appears at 1.45 nm, while that after thermal aging appears at 1.75 nm. The proportion of non-aged soot particles with microcrystalline size below 1 nm and above 3 nm is significantly higher than that of aged soot particles, but the proportion of non-aged soot particles with microcrystalline size between 2 nm and 3 nm is significantly lower than that of aged soot particles. The thermal aging makes both larger and smaller crystallite sizes of basic carbon particles decrease. Fig. 13(c) shows the distribution histogram of the microcrystalline curvature of soot particles. About 54% of non-aged soot particles is greater than 1.2, and this proportion decreases to about 43% after thermal aging. The peak value of microcrystalline curvature of non-aged soot particles appears at 1.25, while the peak value after thermal aging appears at 1.15, and the microcrystalline curvature tends to decrease, which indicates that the structure of soot particles became more orderly.

RETRACTED

**Fig. 13:** Characteristic parameters of non-aged soot particles and soot particles after thermal aging in O_2_/NO_2_ atmosphere: (a) layer spacing; (b) microcrystalline size; (c) microcrystalline curvature.

## Conclusions

In this study, FT-IR and XPS were performed on thermal aging soot samples to investigate the changes in characteristic parameters such as surface functional groups and microstructure of soot. The microstructure and evolution of soot were also analyzed using high magnification lens. The main conclusions are as follows:

(1) Based on the TG analysis results and oxidation kinetics methods of different samples, the activation energy of different soot samples was calculated. The results indicate that the activation energy of thermal aging soot is the highest in N_2_ atmosphere. Under O_2_/NO_2_ atmosphere, the weight loss rate of soot is the highest and the ignition temperature is the lowest. The O_2_ and NO_2_ in the thermal aging atmosphere will cause a decrease in the activation of soot.

(2) The relative content of hydrocarbon functional groups was analyzed based on the FT-IR spectra of different samples. The results showed that the degree and content of hydrocarbon functional group branching decreased after thermal aging. The ratio of *I*_2920_/*I*_2854_ reached the lowest value of 1.19 when the thermal aging atmosphere was NO_2_/O_2_, and the ratio of *I*_2920_/*I*_2854_ reached the lowest value of 0.45 when the atmosphere was O_2_.

(3) Based on the XPS spectra of different samples, the changes in the relative content of oxygen elements and oxygen-containing functional groups on the surface of soot samples were studied. The results indicate that after thermal aging, the surface O element content of soot decreases, and the degree of hybridization of carbon atoms decreases. The content of oxygen-containing functional groups on the surface of thermal aging soot decreased in N_2_ atmosphere. Compared with pure N_2_ atmosphere, the content of C–OH functional groups in soot in O_2_ and O_2_/NO_2_ atmosphere decreased by 11.31% and 10.99%, respectively.

(4) The interlayer spacing, microcrystalline size, and microcrystalline curvature of soot particles were measured using HRTEM, and the changes in the microstructure and graphitization degree of basic carbon particles aged under O_2_/NO_2_ were analyzed. The results show that compared with non-aged soot, the interlayer spacing and microcrystalline curvature of the basic carbon particles in thermal aging soot decrease, the microcrystalline size increases, and the degree of graphitization increases, which is not conducive to the oxidation and combustion of soot.

(5) This study analyzes the process of soot thermal aging based on a thermal aging device platform. Subsequent research can be conducted on the complete DPF carrier structure and actual diesel engine exhaust environment for soot thermal aging experiments. At the same time, performance optimization experiments for DPF regeneration can be conducted based on the research results of soot thermal aging process.

RETRACTED

## Conflicts of interest

There are no conflicts to declare.

## Supplementary Material
